# A Pulmonary Nodule Spiculation Recognition Algorithm Based on Generative Adversarial Networks

**DOI:** 10.1155/2022/3341924

**Published:** 2022-06-24

**Authors:** Jing Zhang, Shi Qiu, Xiaohai Cui, Ting Liang

**Affiliations:** ^1^Department of Thoracic Surgery, The First Affiliated Hospital of Xi'an Jiaotong University, Xi'an, China; ^2^Key Laboratory of Spectral Imaging Technology CAS, Xi'an Institute of Optics and Precision Mechanics, Chinese Academy of Sciences, Xi'an, China; ^3^Department of Radiology, The First Affiliated Hospital of Xi'an Jiaotong University, Xi'an, China; ^4^Department of Biomedical Engineering, The Key Laboratory of Biomedical Information Engineering of the Ministry of Education, School of Life Science and Technology, Xi'an Jiaotong University, Xi'an, China

## Abstract

Pulmonary nodules have been found as the main pathological change in the lung. Signs of pulmonary nodule lay the major basis for the recognition of the benign and malignant of pulmonary nodules. The spiculation of pulmonary nodules is one of the main signs. Pulmonary nodules are small in volume, so they are difficult to extract accurately. Moreover, the number of spiculation samples is limited, so it is difficult to build a stable network structure. Thus, a novel pulmonary nodule spiculation recognition algorithm is proposed. MCA (morphological component analysis) model is built to segment pulmonary nodules in accordance with the composition of pulmonary CT images. Subsequently, the maximum density projection mechanism is introduced to characterize the boundary features of pulmonary nodules to the maximum extent. Inspired by time series dynamic programming, this paper proposes DTW (dynamic time warping) distance to measure data similarity. Lastly, a semisupervised generative adversarial network is built to solve the problem of insufficient positive samples, and it is capable of recognizing pulmonary nodule spiculation. As revealed by the experimental result, the proposed algorithm exhibited strong robustness.

## 1. Introduction

Pulmonary nodule has been found as one type of main diseases in the lung. Malignant pulmonary nodule can be transformed into lung cancer, thus seriously affecting human health [1]. Spiculation lays a solid basis for judging the benign or malignant of pulmonary nodules. The spiculation signs in patients are classified as short or long spiculations. Short spiculation signs take on a critical clinical significance in the diagnosis of peripheral pulmonary cancer [2]. CT has been used as a main method to detect pulmonary nodules [3]. However, the proportion of pulmonary nodules is small in the lung, thus resulting in only limited pixels in CT images, so it is difficult for the detection.

Extensive researches have been conducted on computer-aided diagnosis, and some achievements have been made in the detection of pulmonary nodules, of which several representatives are presented below. Alilou et al. [4] proposed a complete framework for pulmonary nodule detection. Mehta et al. [5] analyzed the correlation between pulmonary nodule volume and benign or malignant. Van Ginneken et al. [6] analyzed the imaging features of pulmonary nodules with a computer. Elsayed et al. [7] proposed an automatic pulmonary nodule detection algorithm. Qiu et al. [8] built a Gestalt model for the detection of pulmonary nodules based on the principle of vision. Dou et al. [9] investigated pulmonary nodules from a 3D perspective. Feng et al. [10] built a CNN network to segment pulmonary nodules. Wilson and Devaraj [11] studied the radiology of pulmonary nodules. Gruetzemacher et al. [12] built a 3D deep learning framework to detect pulmonary nodules. Choi et al. [13] formulated the spiculation quantitative standard of lung cancer. Shen et al. [14] built an international deep hierarchical semantic dynamic network to classify pulmonary nodules. Qiu et al. distinguished between the types of pulmonary nodules [15] by constructing a recurrence plot. Qiu et al. [16] predicted potential burr features through machine learning. Li et al. [17] predicted cancer incidence rate based on burr sign. Marques et al. [18] built multitask CNN to achieve benign and malignant classification of pulmonary nodules. Zhou et al. [19] used a statistical model to predict tumor signs. He et al. [20] proposed an ISHAP-based interpretation model-guided classification method to predict tumor signs. Erdogdu et al. [21] used morphology-isolated pulmonary nodules to predict malignant tumors.

In brief, main detection and sign recognition problems of pulmonary nodules are presented as follows. (1) The boundary of pulmonary nodule is fuzzy, and the membership degree of boundary is not considered in the model, thus causing inaccurate boundary segmentation. (2) The limited feature of pulmonary nodules is observed from one dimension, thus causing inaccurate identification of signs. (3) Due to the limited number of spiculations, the positive and negative samples are not uniform, thus causing poor classification effect.

In this paper, a novel pulmonary nodule spiculation recognition algorithm is proposed based on the above three defects. (1) The model is established based on morphological component analysis to segment pulmonary nodules accurately. (2) A three-dimensional maximum density projection algorithm is proposed to integrate local three-dimensional information into two-dimensional image for the boundary representation of pulmonary nodules. (3) The generative adversarial network based on manifold constraints is built to enhance the stability of sign discrimination.

## 2. Algorithm

The recognition process of pulmonary nodule spiculation is built, as presented in Figure 1. First, MCA (morphological component analysis) model is established to segment pulmonary nodules. Then, the maximum density projection model is established from axial, coronal, and sagittal planes to characterize the boundary of pulmonary nodules. The boundary is expanded into time series, and DTW (dynamic time warping) algorithm is adopted to measure the similarity between the sample and the database for the spiculation recognition. To solve the problem of imbalance between positive and negative samples, an adversarial network based on manifold constraint is built. A complete recognition process of pulmonary nodule spiculation is established.

### 2.1. Segmentation Algorithm Based on Morphological Component Analysis

One pulmonary CT image **I** comprises pulmonary nodule **I**_*o*_, tissue area **I**_*s*_, and background **I**_*b*_.

(1) $$\begin{array}{c} I=I_{o}+I_{s}+I_{b}. \end{array}$$

Pulmonary nodules are locally highlighted with limited pixels in CT images, as presented in Figure 2. The complete segmentation of pulmonary nodules is the premise of pulmonary nodule sign recognition.

In accordance with the analysis of CT composition of lung, morphological component analysis (MCA) is introduced to segment **I**_*s*_ [22]. MCA suggests that the signal comprises a series of component signals. The respective morphological component exhibits a unique dictionary sparsity corresponding to it. Accordingly, different signal components can be identified by dictionary.

Then, **I** can be represented by *K* morphological components:

(2) $$\begin{array}{c} I=\overset{3}{\underset{k=1}{\sum }}I_{k}=\overset{3}{\underset{k=1}{\sum }}D_{k}\alpha_{k}, \end{array}$$

where **D**_*k*_ denotes a super complete dictionary and *α*_*k*_ represents the sparse coefficient. In the solving process, the solution of the equation is not unique since the limit that the number of unknown parameters is greater than the number of equations. To ensure the sparsity maximization, MCA model is established:

(3) $$\begin{array}{c} \begin{array}{c} \underset{\alpha_{1},..\alpha_{3}}{\min}\overset{3}{\underset{k=1}{\sum }}{\left\|\alpha_{k}\right\|}_{p}\\ s.t.{\left\|I-\overset{3}{\underset{k=1}{\sum }}D_{k}\alpha_{k}\right\|}_{2}\leq \Gamma . \end{array} \end{array}$$

where Γ represents the error between the original signal and the combined classification and ||.||*_p_* is *p* norm.

Since there is a significant difference among **I**_*o*_, **I**_*s*_, and **I**_*b*_, and pulmonary nodules cannot be in the range of **I**_*b*_, only **I**_*o*_ and **I**_*s*_ are calculated by MCA model:

(4) $$\begin{array}{c} \left\{\begin{array}{cc} \alpha_{o}=\arg\min{\left\|\alpha_{o}\right\|}_{0} & s.t.I_{o}=D_{o}\alpha_{o},\\ \alpha_{s}=\arg\min{\left\|\alpha_{s}\right\|}_{0} & s.t.I_{s}=D_{s}\alpha_{s}. \end{array}\right. \end{array}$$

The optimization problem is then transformed into

(5) $$\begin{array}{c} \begin{array}{c} \left\{\alpha_{o}^{opt},\alpha_{s}^{opt}\right\}=\arg\min\left({\left\|\alpha_{o}\right\|}_{0}+{\left\|\alpha_{s}\right\|}_{0}\right),\\ s.t.{\left\|I-D_{o}\alpha_{o}-D_{s}\alpha_{s}\right\|}_{2}\leq \delta . \end{array} \end{array}$$

It is to find the sparse representation of the signal from the super complete dictionary, and its computational complexity increases with the increase in the number of dictionary columns. According to the BP algorithm, norm *L*0 in the equation can be replaced by norm *L*1, and then, Equation (5) becomes a linear programming problem:

(6) $$\begin{array}{c} \left\{\alpha_{o}^{\text{opt}},\alpha_{s}^{\text{opt}}\right\}=\arg\min\left({\left\|\alpha_{o}\right\|}_{1}+{\left\|\alpha_{s}\right\|}_{1}\right)+\lambda {\left\|I-D_{o}\alpha_{o}-D_{s}\alpha_{s}\right\|}_{2}+\gamma V\left(D_{o}\alpha_{o}\right). \end{array}$$

where *λ* and *γ* are the weights and *V* is the total change of pulmonary nodules.

As revealed by the above analysis, the extraction of dictionary is of great significance. Curvelet transform is adopted to sparsely represent the smooth part of the image, and local discrete cosine transform is employed to represent the texture part of the image.

Curvelet transform [23] represents the anisotropic elements in the image and better expresses the image edge, and the definition is as follows:

(7) $$\begin{array}{c} C\left(j,l,k\right)=\int_{R^{2}}I\left(x,y\right)\varphi_{j,l,k}dxdy, \end{array}$$

where *C*(*j*, *l*, *k*) is the curvelet transform coefficient and *φ*_*j*,*l*,*k*_ is the wavelet basis.

Local discrete cosine transform (LDCT) can represent the component of texture in image, as defined below:

(8) $$\begin{array}{c} \begin{array}{c} C\left(u,v\right)=a\left(u\right)a\left(v\right)b\left(u,v\right),\\ b\left(u,v\right)=\overset{M-1}{\underset{x=0}{\sum }}\overset{M-1}{\underset{y=0}{\sum }}I\left(x,y\right)\cos\left[\frac{\left(2x+1\right)u\pi }{2M}\right]\cos\left[\frac{\left(2y+1\right)v\pi }{2N}\right], \end{array} \end{array}$$

where *C*(*μ*, *v*) denotes the discrete cosine transform coefficient.

Based on the decomposition of MCA algorithm, the threshold segmentation algorithm is employed to extract the pulmonary nodule region.

(9) $$\begin{array}{c} \left\{D_{o}^{opt},D_{s}^{opt}\right\}=\arg\min\left({\left\|D_{o}^{*}I_{o}\right\|}_{1}+{\left\|D_{o}^{*}I_{o}\right\|}_{1}\right)+\lambda {\left\|I-I_{o}-I_{s}\right\|}_{2}+\gamma V\left(I_{o}\right), \end{array}$$

(10) $$\begin{array}{c} D^{*}=D^{T}{\left({DD}^{T}\right)}^{-1}. \end{array}$$

**α**_*o*_^∗^ is selected from **α**_*o*_ to reconstruct the image

(11) $$\begin{array}{c} I_{o}=D_{o}^{\text{opt}}\alpha_{o}^{*}. \end{array}$$

The watershed algorithm is applied. Set *C*(*M*_*i*_) as the catchment basin in the minimal area *M*_*i*_ related, and *T*[*n*] denote the set of points satisfying the condition *g*(*x*, *y*) < *n*. According to

(12) $$\begin{array}{c} \begin{array}{c} C_{n}\left(M_{i}\right)=\left\{\begin{array}{cc} 1, & C\left(M_{i}\right)\cap T\left[n\right],\\ 0, & \text{others}, \end{array}\right.\\ T\left[n\right]=\left\{\left(x,y\right)\left|g\left(x,y\right)\leq n\right.\right\}. \end{array} \end{array}$$

The image after segmentation can be obtained. To enhance the boundary signal intensity of pulmonary nodules, a rectangular region is selected for the region where pulmonary nodules are located. The gradient transformation is used as input:

(13) $$\begin{array}{c} G_{o}\left(x,y\right)=\sqrt{{\left(\frac{\partial I_{o}\left(x,y\right)}{\partial x}\right)}^{2}+{\left(\frac{\partial I_{o}\left(x,y\right)}{\partial y}\right)}^{2}}. \end{array}$$

Morphological open and close operation is applied to the gradient image to remove some redundant local minimum areas. The next step is to locate the local minimum pixel and its adjacent region. Lastly, the gradient image is applied twice by the watershed algorithm to obtain the region of pulmonary nodules.

### 2.2. Multidirection Projection Sign Analysis Algorithm

Pulmonary nodules have 3D tissue structure. However, when extracting from the conventional axial direction, pulmonary nodules can lead to incomplete burr information. However, 3D pulmonary nodule model has a large amount of calculation, which cannot meet the demand of real-time detection [24]. Thus, the concept of maximum density projection is introduced:

(14) $$\begin{array}{c} M\left(x,y\right)=\max\left(I_{0}\left(x,y\right)\cdots I_{N}\left(x,y\right)\right). \end{array}$$

The local 3D information of pulmonary nodules can be displayed from one location. However, only from the MIP projection image of a single position, the spiculation perpendicular to the projection plane can submerge into the MIP image, as presented in Figure 3. Accordingly, we build a multidirectional MIP density projection algorithm to ensure that any spiculation is not missed.

According to the definition of spiculation, physicians mainly distinguish by observing the boundary characteristics of pulmonary nodules. It is necessary to choose an appropriate algorithm to analyze the boundary of pulmonary nodules. Conventional statistical analysis methods are based on the assumption that the data sequence has independence. Time series analysis [25] is different from conventional statistical methods, which focuses on the study and analysis of the interdependence of data series. Thus, in this paper, we take the center of the pulmonary nodule as the center of the circle (*x*_0_, *y*_0_) and the boundary closest to (*x*_0_, *y*_0_) as the starting point to expand the MIP images in different directions clockwise to form a time series for analysis, as presented in Figure 4.

(15) $$\begin{array}{c} \left\{\begin{array}{c} \rho =\sqrt{{\left(x-x_{o}\right)}^{2}+{\left(y-y_{o}\right)}^{2}},\\ \theta =\arctan\frac{y-y_{o}}{x-x_{o}}. \end{array}\right. \end{array}$$

According to the definition of spiculation, the spicule area of protuberance is only considered, instead of the flat area [26]. For this reason, we extract the protuberance regions from the unfolded image and sort them into a new time series according to the degree of protuberance for analysis.

The sequence is compared with the trained data in the database to determine whether it is the spiculation. The DTW distance of dynamic programming is introduced based on the scalability of time series to measure the degree of data similarity [27].

(16) $$\begin{array}{c} \left\{\begin{array}{c} D\left(P,Q\right)=f\left(n,m\right),\\ f\left(n,m\right)=d\left(P_{i},Q_{i}\right)+\min\left(f\left(i,j-1\right),f\left(i-1,j\right),f\left(i-1,j-1\right)\right),\\ f\left(0,0\right)=0,f\left(0,i\right)=f\left(j,0\right)=\infty , \end{array}\right. \end{array}$$

where *d*() denotes Euclidean distance. The schematic diagram of DTW distance is illustrated in Figure 5. Signs of pulmonary nodules are distinguished according to the degree of similarity.

### 2.3. Semisupervised Generative Adversarial Network

During pulmonary nodule classification, the amount of spiculation data is less than the total number of pulmonary nodules. To solve the problem of uneven distribution of samples, scholars have proposed an unsupervised generative model based on Game Theory (GAN), as presented in Figure 6.

The model consists of generator *A* and discriminator *B*. The optimization process is the training process of binary minimax confrontation. The objective function is

(17) $$\begin{array}{c} \underset{A}{\min}\underset{B}{\max}V\left(A,B\right)=E\left(\log A\right)+E\left(\log\left(1-B\right)\right). \end{array}$$

To apply GAN to semisupervised learning, it is assumed that classifier *H*_*θ*_ output *k*-dimensional vector *l* = {*l*_1_, *l*_2_, ⋯*l*_*K*_}, and generate output probability through softmax function

(18) $$\begin{array}{c} P\left(y=i\left|x\right.;\theta \right)=\frac{\exp l_{i}\left(x\right)}{\sum_{k=1}^{K}\exp l_{k}\left(x\right)}, \end{array}$$

where *P*(*y* = *i*|*x*; *θ*) denotes the probability that the real sample *x* belongs to class *I*. Discriminator *B*_*θ*_ is adopted to distinguish the real sample *x* from the generated sample *x*_*g*_:

(19) $$\begin{array}{c} B_{\theta }\left(x\right)=\frac{\sum_{k=1}^{K}\exp l_{k}\left(x\right)}{1+\sum_{k=1}^{K}\exp l_{k}\left(x\right)}. \end{array}$$

The loss function is yielded as

(20) $$\begin{array}{c} L=E\left[\log\left(1+\overset{K}{\underset{i=1}{\sum }}\exp l_{i}\left(x_{g}\right)\right)\right]-E\left[\log\overset{K}{\underset{i=1}{\sum }}\exp l_{i}\left(x\right)-\log\left(1+\overset{K}{\underset{i=1}{\sum }}\exp l_{i}\left(x\right)\right)\right]. \end{array}$$

The derivation of *L* is as follows:

(21) $$\begin{array}{c} \nabla L=E\left[\overset{K}{\underset{i=1}{\sum }}P\left(y=i\left|x_{g}\right.\right)\nabla l_{i}\left(x_{g}\right)\right]-E\left[\overset{K}{\underset{i=1}{\sum }}\left\{P\left(y=i\left|x\right.,y\leq K\right)-P\left(y=i\left|x\right.\right)\right\}\nabla l_{i}\left(x\right)\right]. \end{array}$$

To ensure *L* minimization, the updating process will promote the network to further enhance the current prediction *P*(*y* = *i*|*x*; *θ*). At the same time, the activation value of the predicted class connected neurons will be updated to the maximum, so the false prediction will be enhanced by map updating to get worse enhancement.

The classifier exhibiting better classification performance is obtained by considerable editing training samples at the early stage or by fully learning at the later stage. If the classifier is not mature and the resolution is not strong, it will produce wrong prediction. This problem will be reflected in the task of using a small number of labeled samples. Especially at the early stage of learning, the classifier is too poor to show enough discriminative power on the above samples.

Accordingly, the discriminator *B* is optimized by variable loss rather than the original counter loss. The update of the network at the early stage of training does not depend on the prediction of the classifier, and the standard deviation matching loss in the generator is introduced to stabilize the GAN training. To optimize the performance of the classifier, manifold regularization term which is convenient for GAN calculation is added to the variable loss to further increase the robustness of the classifier to manifold local disturbance.

First, we improve the discriminator to alleviate the adverse effects of poor classifiers at the early stage of training on a small number of labeled samples:

(22) $$\begin{array}{c} B_{\theta }^{*}\left(x\right)=\frac{\exp\left(\left(1/K\right)\sum_{k=1}^{K}l_{k}\left(x\right)\right)}{1+\exp\left(\left(1/K\right)\sum_{k=1}^{K}l_{k}\left(x\right)\right)}, \end{array}$$

where *B*_*θ*_^∗^ is to distinguish the real image and generate the image based on the mean value of the activation value of the last layer *K* neurons. *B*_*θ*_^∗^ is updated to

(23) $$\begin{array}{c} \left\{\begin{array}{c} -\frac{\partial \left[-\log\left\{B_{\theta }^{*}\left(x\right)\right\}\right]}{\partial l_{i}\left(x\right)}=\frac{1}{K}P\left(fake\left|x\right.;B_{\theta }^{*}\right),\\ -\frac{\partial \left[-\log\left\{1-B_{\theta }^{*}\left(x_{g}\right)\right\}\right]}{\partial l_{i}\left(x_{g}\right)}=-\frac{1}{K}P\left(real\left|x_{g}\right.;B_{\theta }^{*}\right). \end{array}\right. \end{array}$$

The above neurons are only activated on the real image *x* to form the subspace of the feature *l*_*i*_(*x*) of the real image. Since the generator provides a more realistic generated image *x*_*g*_, the subspace becomes more compact to facilitate the classifier learning, and the focus is placed on the labeled samples in the limited subspace to facilitate the generalization of the classifier on it.

Discriminator *B*_*θ*_^∗^ is capable of effectively solving the problem of poor performance of the previous classifiers by not relying on the current prediction. However, for the classifiers with good classification performance in the middle and later learning stages, *B*_*θ*_ can be employed to replace them.

Manifold regularization term is introduced to increase the robustness of the classifier to local disturbances. For classifiers *φ*_*θ*_, ▽_*z*_*φ*_*θ*_(*B*(*z*^(*i*)^)) expresses the change of classification decision on manifold formed by *B*(*z*^(*i*)^), and the change of *φ*_*θ*_ restricted by *B*(*z*^(*i*)^) is written as

(24) $$\begin{array}{c} {\left\|\varphi_{\theta }\left(G\left(z^{\left(i\right)}+\delta \right)\right)-\varphi_{\theta }\left(G\left(z^{\left(i\right)}\right)\right)\right\|}^{2}\approx {\left\|\nabla_{z}^{g}\varphi_{\theta }\left(G\left(z^{\left(i\right)}\right)\right)\right\|}^{2}\delta z, \end{array}$$

where ∇_*z*_^*g*^*φ*_*θ*_(*G*(*z*^(*i*)^)) is capable of training the classifier to resist the small disturbance on the manifold, ‖∇_*z*_^*g*^*φ*_*θ*_(*G*(*z*^(*i*)^))‖^2^*δz* is adopted to approximate the regular term of the manifold, and *ξ* is employed to adjust the step size of updating the gradient direction of the manifold:

(25) $$\begin{array}{c} \Psi \left(\varphi_{\theta }\right)=\frac{1}{n}\overset{n}{\underset{i=1}{\sum }}{\left\|\varphi_{\theta }\left(G\left(z^{\left(i\right)}+\frac{\varepsilon \delta }{\left\|\delta \right\|}\right)\right)-\varphi_{\theta }\left(G\left(z^{\left(i\right)}\right)\right)\right\|}^{2}. \end{array}$$

The loss function of discriminator is written as

(26) $$\begin{array}{c} \left\{\begin{array}{c} \underset{\theta }{\min}L=\alpha L_{1}+\beta L_{2}+\gamma \Psi \left(\varphi_{\theta }\right)\text{: }\;\alpha +\beta +\gamma =1,\\ L_{1}=E\left[-\log\left\{P\left(y=i\left|x;\theta \right.\right)\right\}\right],\\ L_{2}=E\left[-\log\left\{B_{\theta }^{*}\left(x;w\right)\right\}\right]+E\left[-\log\left\{1-B_{\theta }^{*}\left(x_{g};w\right)\right\}\right], \end{array}\right. \end{array}$$

where *α* represents the weight coefficient of supervision loss, *Β* represents the weight coefficient of unsupervised loss, and *γ* represents the manifold regular term weight coefficient.

To improve the stability of training GAN, the standard deviation matching loss is introduced:

(27) $$\begin{array}{c} \underset{\eta }{\min}L={\left\|\mu_{\theta }^{l}-\mu_{\theta ,\eta }^{l}\right\|}^{2}+{\left\|\sigma_{\theta }^{l}-\sigma_{\theta ,\eta }^{l}\right\|}^{2}, \end{array}$$

where *μ*_*θ*_^*l*^, *μ*_*θ*,*η*_^*l*^, *σ*_*θ*_^*l*^, and *σ*_*θ*,*η*_^*l*^ denote the mean and standard deviation of the real and generated images in the classifier output vector, respectively.

## 3. Experiment and Result Analysis

The experimental data were acquired from the international early lung cancer action project and the American lung imaging association database [28]. A total of 514 pulmonary nodule spiculation and 501 nonpulmonary nodule spiculation were labeled by two professional doctors as the basis of algorithm detection. CT data were 16 bits. The window width was adjusted to 1250~1600 HU to more effectively observe pulmonary nodules. It was normalized to [0,1] within the above range. The input image was normalized to 512 × 512.

### 3.1. Image Segmentation

To verify the performance of the proposed algorithm, the following indicators are introduced for measurement [15]:

(28) $$\begin{array}{c} \left\{\begin{array}{c} \text{AOM}=\frac{R_{s}\cap R_{g}}{R_{s}\cup R_{g}},\\ \text{AVM}=\frac{R_{s}-R_{g}}{R_{s}},\\ \text{AUM}=\frac{R_{g}-R_{s}}{R_{g}},\\ CM=\frac{1}{3}\left\{\text{AOM}+\left(1-\text{AVM}\right)+\left(1-\text{AUM}\right)\right\}, \end{array}\right. \end{array}$$

where *R*_*g*_ denotes gold standard, *R*_*s*_ represents segmentation results, AOM and CM are proportional to the segmentation result, and AVM and AUM are inversely proportional to the segmentation results.

The segmentation effect of different algorithms was compared. As depicted in Table 1, Reference [9] built the model from 3D perspective to extract the overall structure of pulmonary nodules, and the built model is capable of achieving better segmentation of pulmonary nodules. Reference [10] built CNN network using a deep learning method to segment single-layer pulmonary nodules. Reference [29] combined watershed with pixel attribution probability to develop a network for the segmentation of pulmonary nodules. Reference [30] built the dual-branch residual network by fusing the whole and local information of the image for the segmentation of pulmonary nodules. The proposed algorithm is adopted to build the MIP model in accordance with three positions. It fuses the three-dimensional information into the local image and then uses the segmentation algorithm based on morphological component analysis to achieve effective results.

### 3.2. Multidirection MIP Algorithm Effect

To verify the effectiveness of the algorithm, the detection rate for measurement is presented.

(29) $$\begin{array}{c} F=\frac{A}{B}. \end{array}$$

The coronal and sagittal images were reconstructed in accordance with the CT axial images, and the axial, coronal, and sagittal images with the most obvious characteristics of pulmonary nodules were selected, respectively, for the comparison with the MIP algorithm, as listed in Table 2. It is not comprehensive to observe the signs of pulmonary nodules from a single location, which cannot indicate the overall characteristics of pulmonary nodules. With the increase in observation angles, the manifestation of pulmonary nodules increases to 92%. The MIP algorithm fuses local information into MIP image, which can show local 3D information, and significantly increases the detection rate of single position in a single frame. The detection rate of MIP algorithm can reach 98%, whereas there are still a few pulmonary nodule spiculation syndrome that are not detected, which is primarily because the segmentation is missed.

As depicted in Figure 7, the common pulmonary nodule (Figure 7(a)) is round in axial, coronal, and sagittal images. The boundary is smoother. In Figure 7(b), the type of pulmonary nodule with vascular adhesion is round in axial view and radial in coronal and sagittal view. If only from the axis detection, there will be the risk of missing detection. The internal structure of MIP can be displayed more intuitively through the three positions of MIP. In Figure 7(c), the features of spiculation are not obvious in axial, coronal, and sagittal view. After MIP, the local 3D information is fused into the image to get the intuitive spiculation structure. It lays a foundation for the recognition of spiculation feature.

### 3.3. Recognition Algorithm of Spiculation

The features extracted in this paper are intuitively presented in Figure 8. First, the MIP image of pulmonary nodules is expanded from the axial, coronal, and sagittal planes to the same coordinate system. Subsequently, the lowest point of the respective position is determined as the benchmark for removal to obtain the spiculation features. As depicted in Figure 8(a), the depression of common pulmonary nodules is small, and the boundary is relatively smooth, so more region is removed. Boundary of spiculation pulmonary nodule in Figures 8(b) and 8(c) is relatively steep, so the removal is relatively less. As a result, the accurate recognition of pulmonary nodules is achieved.

Since there are fewer positive samples and more negative samples in the identification process of pulmonary nodules, the following indicators are introduced to evaluate the performance of the algorithm:

(30) $$\begin{array}{c} \left\{\begin{array}{c} \text{SEN}=\frac{\text{TP}}{\text{TP}+\text{FN}},\\ \text{SPE}=\frac{\text{TN}}{\text{TN}+\text{FP}},\\ \text{ACC}=\frac{\text{TP}+\text{TN}}{\text{TP}+\text{FP}+\text{TN}+\text{FN}},\\ \text{FPF}=1‐\text{ACC}, \end{array}\right. \end{array}$$

where TP denotes true positive, FP represents false positive, FN is false negative, and TN is true negative. The results are listed in Table 3. SVM [4] algorithm is adopted to build linear classifiers for classification. DTW [27] algorithm uses the sequence correlation to set thresholds to achieve classification. CNN [10] algorithm is adopted to build a convolutional neural network for developing the correlation between pixel value and target and realize classification. The semisupervised generative adversarial network proposed in this paper comprehensively considers the correlation between positive samples and negative samples, thus improving the loss function and leads to good results.

To verify the proposed algorithm for spiculation recognition, ROC curves are introduced to measure its effect. As depicted in Figure 9, ROC curves indicate the results of axial, coronal, and sagittal positions, suggesting that the ability to extract pulmonary nodules from axial position is limited. With the increase in observation locations, the extraction performance of pulmonary nodules tends to increase, and the effect is optimal at three positions.

Reference [14] proposed an interpretable deep hierarchical semantic convolutional neural network (IDHSCNN) to fuse semantic information into images for the recognition of different signs. In Reference [16], deep learning (DL) is adopted to analyze the single-layer pulmonary nodules and identify the signs. In Reference [31], the shape feature is employed to classify pulmonary nodules. In Reference [32], pulmonary nodule signs are identified based on edge gradient (EG) information. The above algorithms are adopted to build models for recognizing pulmonary nodules from different perspectives. However, the problem of limited feature samples is not considered, so the improvement is not significant in large samples. The semisupervised generative adversarial network proposed reduces the imbalance of positive and negative samples while achieving a better recognition effect

## 4. Conclusion

Pulmonary nodule spiculation is difficult to segment and recognize. To solve this problem, a segmentation algorithm based on morphological component analysis is proposed by focusing on the intrinsic features of pulmonary nodules. A multidirection MIP algorithm is proposed to solve the problems of inaccurate representation of single position and complex 3D modeling, which fuses multidirection information to accurately represent pulmonary nodules. To solve the problem of poor network stability caused by the imbalance of positive and negative samples, a semisupervised generative adversarial network is proposed to increase the recognition rate of pulmonary nodule spiculation. In future research, research on computer-aided detection of pulmonary nodules should be conducted to enhance the ability of automatic detection of pulmonary nodules. The characteristics exhibited by COVID-19 will be explored, and novel pneumonia detection and recognition systems will be developed.

## Figures and Tables

**Figure 1:** Recognition process of pulmonary nodule spiculation.

**Figure 2:** Gray scale image of a pulmonary nodule.

**Figure 3:** Multidirectional MIP effect.

**Figure 4:** Boundary unfolding of pulmonary nodules.

**Figure 5:** DTW distance.

**Figure 6:** Network structure.

**Figure 7:** Multidirection MIP images of pulmonary nodule.

**Figure 8:** Computer features of spiculation.

**Figure 9:** ROC curve.

**Table 1:** Comparisons of image segmentation algorithms.

Algorithm	AOM	AVM	AUM	CM
3D	0.78	0.31	0.29	0.73
CNN	0.71	0.35	0.33	0.68
Watershed	0.75	0.33	0.31	0.7
DBRN	0.80	0.26	0.27	0.76
Ours	0.83	0.22	0.20	0.80

**Table 2:** Comparison of algorithm effect.

Algorithm	*F*	
	Normal	MIP
Axial	80	91
Coronal	82	90
Sagittal	80	90
Multidirectional	92	98

**Table 3:** Detection effect.

Algorithm	SEN	SPE	ACC	FPF
SVM	81	12	85	15
DTW	86	10	89	11
CNN	90	6	91	9
Ours	94	4	93	7

## Data Availability

Data are available from the International Early Lung Cancer Action Project (http://www.via.cornell.edu/lungdb.html).
